The article "Application of CT Scan in Diagnosis of Iliac-Femoral Vein Thrombosis after Hip Replacement" was retracted in 2023. Reasons: signs of a paper mill; suspected computer-generated content; unreliable results or conclusions; lack of ethics approval or compliance.

# Application of CT Scan in Diagnosis of Iliac-Femoral Vein Thrombosis after Hip Replacement

**DOI:** 10.1155/2022/8428963

**Published:** 2022-06-20

**Authors:** Dong Li, Lishan Wang, Zhanxin Li, Libin Li, Qingwei Wang, Li Zhang, Zhigang Guo

**Affiliations:** ^1^North China Medical&Health Group Xingtai General Hospital, Xingtai, Hebei 054000, China; ^2^Respiratory Department of Hebei General Hospital for Veterans, Xingtai, Hebei 054000, China

## Abstract

Based on the knowledge of the previous film, the CT scan was used to diagnose the disease of women and men after the diagnosis of atherosclerosis by scanning the CT microscope. This article first examines the existing medical procedures in China, highlighting the advantages and disadvantages of various systems in terms of usability and user experience. Combined with the actual needs of hospitals, this paper developed a set of preoperative intelligent measurement system (MIPS) based on pattern recognition for total skeletal joint replacement. It is beneficial for doctors to better observe the lesions of patients before surgery and carry out necessary operations in the PATIENT DR film. In the process, the model is used to identify the patient, and the patient is given a fake score based on the characteristics of the DR film. In nonsymptomatic patients, 13.5% had muscle contraction > 50%, 2.0% had muscle contraction 70%, and the mean pelvic area was 23.48%. The left ventricular muscle has a 45.0% contraction rate, the left ventricle has a 70% contraction, and the median contraction rate is 47.58%. The right muscle, which is inserted between the right artery and the inner lymphatic artery, is the most common type of compression of the right muscle, accounting for 59.26%. In terms of the mean muscle contraction rate on the right side, patients with DVT with right muscles were higher than patients with DVT with left ventricles (48.54% to 22.29%, *P* < 0.001). The mean incidence of left ventricular DVT patients was higher than that of right ventricular DVT patients (71.88% versus 45.83% *P* < 0.0011).

## 1. Introduction

At present, China has a certain theoretical basis for the study of deep vein thrombosis after bone joint replacement and some prevention systems, but most of them are clinical experience, and there is a lack of clinical application standards based on evidence-based theory for the prevention of deep vein thrombosis. Nursing managers and clinical nursing workers in China are focusing on the appropriate prevention measures and effects of DVT, but the viewpoints are outdated and the content is relatively limited. More importantly, current studies lack evidence-based prevention strategies and cluster interventions for DVT, as well as simple, scientific, and effective guiding prevention measures and standardized standards in clinical work, which are not conducive to nursing quality management and process monitoring. In 2008, the American College of Chest Physicians (ACCP) has developed the 8th edition of its clinical practice guidelines for antithrombotic therapy and thrombotic prophylaxis and issued the 9th edition in 2012. Evidence-based nursing (EBN) is a nursing concept, which is influenced by evidence-based medicine (EBM), also known as evidence-based nursing. The core idea of evidence-based nursing is to use the most reliable scientific evidence to achieve the best nursing effect, which contains three elements: first, use the most appropriate nursing research evidence; second, the clinical experience and personal skills of the nursing staff; and third, the patient's actual situation, values, and subjective will. Combine these three elements together to guide practical work. The implementation of nursing for patients should be patient-centered and should also be combined with the personal experience and rich clinical skills of nursing staff.

The article "Application of CT Scan in Diagnosis of Iliac-Femoral Vein Thrombosis after Hip Replacement" was retracted in 2023. Reasons: signs of a paper mill; suspected computer-generated content; unreliable results or conclusions; lack of ethics approval or compliance.

## 2. Literature

Gitelzon et al. said that in recent years, with the rapid development of expressways and railways, cars and electric vehicles have increased dramatically, and people's lifestyles have changed. These factors lead to an increase in the incidence of car accidents, joint injury and joint disease, and the deterioration of patients' joint function, leading to the reduction of patients' quality of life [1]. Is et al. said a study shows that joint replacement is on the rise, increasing by 11 percent a year in Europe and the United States and in China, too [2]. Ming et al. said that the patient's damaged limb joints cannot be repaired and replaced with prosthetic limbs, which are usually made of artificial materials to replace the damaged joints, so as to restore and improve the structure and function of the affected joints [3]. At present, total skeletal joint replacement is effective and widely used. Lm et al. said that artificial joint replacement has the advantages of relieving pain, maintaining joint stability, improving joint movement, and preventing shortened and deformed limbs [4]. But artificial joint replacement is not perfect. Dozie et al. said that in addition to the limitation of the stability of the joint itself, venous thromboembolism (VTE) and potentially more harmful secondary pulmonary embolism (PTE) have been widely concerned with the widespread development of such surgeries [5]. One study showed that in patients undergoing joint replacement surgery without effective anticoagulant therapy, many patients developed thrombosis after surgery, and the incidence of deep vein thrombosis reached 88,070. Even with effective interventions, the incidence is high, with approximately 2% to 5% of patients presenting with symptoms of VTE. In the United States, approximately 300,000 people die from DVT each year. Deep vein thrombosis kills about 300,000 people a year in the United States. Zhang et al. said that DVT can cause swelling, pain, and even necrosis of the affected limb, requiring amputation in severe cases, significantly reducing the ability to work and quality of life. More importantly, thromboembolism can be secondary to pulmonary embolism, which can even lead to death due to the urgency and severity of the disease [6]. Therefore, in the diagnosis, treatment and nursing work of joint replacement, prevention, and effective intervention should be strengthened. The patient underwent bone joint replacement surgery and developed deep vein thrombosis after surgery, mainly due to the slow blood flow of the three elements of thrombosis (identified by Virchow in 1856): the main causes of slow blood flow are the weakening of local venous return power caused by the lack of muscle pump in the affected limbs and the weakening of systemic venous return power caused by systemic cardiac function. Popivanov et al. said that due to the need to use anesthesia and sedative muscle relaxation drugs during the operation of the patient, at the same time, the postoperative limb needs a longer time to brake, which better provide local stability for fracture healing, resulting in temporary partial or complete loss of muscle pump function, and local venous return power weakened and slowed down [7]. When the patient's systemic blood flow slowed down and local affected limb blood flow slowed down, local tissues appeared metabolic waste retention, different degrees of tissue hypoxia, and some cell metabolism abnormalities. This can not only lead to decreased fibrinolytic activity and local thrombin aggregation but also lead to varying degrees of vascular endothelial damage, thereby promoting local venous thrombosis. Damage to the blood vessel wall: the normal lining of blood vessels is a barrier to platelet aggregation. Endothelial cells produce prostaglandins, a hormone that dilates blood vessels. In the process of artificial bone arthroplasty, although the adjacent blood vessels are rarely directly damaged, they can still be indirectly damaged. The main possibilities are as follows: indirect injury of bone cement during surgery, thermal injury, infection, and chemical injury. Gitelzon et al. said that the thermal effect of cement can cause blood vessel damage and exogenous clotting when it is filled with cement [1]. In addition, the above mentioned local tissue metabolic waste retention of different degrees of hypoxia and abnormal cell metabolism caused by local and systemic slow blood flow of the affected limb can also lead to intima vein injury. Hypercoagulable state: increased clotting factors can increase blood viscosity. For patients undergoing artificial bone arthroplasty, stimulating cytokines released by local injury and systemic stress response can lead to increased clotting factors, inactivation of fibrinolytic system, and thrombosis. In the process of coagulation fibrinolysis and thrombosis, D dimer changes and can reflect fibrinolysis activity, so DD can be used as a test indicator for diagnosis and monitoring of thrombosis. Yadavalli et al. said that there are many factors that can affect the formation of blood clots during bone arthroplasty [8]. These factors include reduced preoperative activity, immobilization, prolonged postoperative bed rest, and the administration of a tourniquet, which may slow venous return. Stress response surgical trauma, thermal injury of local tissue caused by bone cement, and mannitol used to relieve postoperative soft tissue swelling can cause intima injury. At last, perioperative blood loss, fasting, and abstaining from drinking may result in blood concentration and hypercoagulability due to volume factors. Therefore, skeletal joint replacement is a high-risk disease for DVT. Salahuddin and Armstrong said that risk factors for DVT include advanced age, bed rest after trauma, anesthesia, foreign body implantation, and a history of blood clots [9]. In patients with deep vein thrombosis, there are many clinical symptoms. For example, lower limbs can appear pain swelling, skin pigmentation, skin sclerosis, venous ulcer, and so on. Patients even lose the labor force, increasing the pain and economic burden of patients. Therefore, the focus of DVT treatment is prevention. We should do a good job in the assessment of high-risk factors and actively take scientific and reasonable treatment and nursing methods for effective preventive intervention. See Figure 1.

The article "Application of CT Scan in Diagnosis of Iliac-Femoral Vein Thrombosis after Hip Replacement" was retracted in 2023. Reasons: signs of a paper mill; suspected computer-generated content; unreliable results or conclusions; lack of ethics approval or compliance.

## 3. Method

The UI is also known as the user interface, which is between the system and the user, which knows the internal information and allows people to take the form of the user interface and interact between the user and the device. The related software designed for mutual interaction and communication enables users to operate the hardware conveniently and effectively to achieve two-way interaction and complete the desired work. This will make it easier for users to complete the hardware and successfully complete the interface and on-demand tasks. The user interface is broadly defined, including human-computer interaction and graphical user interface. The user interface exists in the field of human and mechanical information exchange [10]. In the long history of interface design and software development, he has been called an artist who does not pay attention to the work of interface design and insults people. In fact, the design of the software interface is similar to the standard design of commercial products, which is the key to purchasing. Interface design is not an easy artwork, it needs to locate the use of the user environment and design for the end user. Therefore, the design of the interface should be combined with user research, which is the process of creating a visual experience for end users [11]. Critically speaking, the interface can be divided into two levels: cognitive (visual, visual, and auditory) and cognitive. The user interface design is an important part of the test equipment [12, 13]. Interface design is a complex task that involves many disciplines such as thinking, reasoning, and speaking, in which everyone plays an important role. The three principles of user interface design are as follows: put the interface under the control of the user; reduce the memory burden of users; keep the interface consistent. Image translation is one of the simplest geometric transformations. Image translation means that all points in the image are blown horizontally and vertically according to the specified translation amount. Let (*x*_0_, *y*_0_) be a point on the original image, the horizontal translation of the image is *t*_*x*_, and the vertical translation is *t*_*y*_; then, the coordinates of the point (*x*_0_, *y*_0_) after the translation will become (*x*_1_, *y*_1_). Obviously, the relationship between (*x*_0_, *y*_0_) and (*x*_1_, *y*_1_) is shown in

(1) $$\begin{array}{c} \left\{\begin{array}{c} x_{1}=x_{0}+t_{x},\\ y_{1}=y_{0}+t_{y}. \end{array}\right. \end{array}$$

The matrix representation is shown in

(2) $$\begin{array}{c} \left[\begin{array}{c} x_{1}\\ y_{1}\\ 1 \end{array}\right]=\left[\begin{array}{ccc} 1 & 0 & t_{x}\\ 0 & 1 & t_{y}\\ 0 & 0 & 1 \end{array}\right]\left[\begin{array}{c} x_{0}\\ y_{0}\\ 1 \end{array}\right]. \end{array}$$

The inverse of the matrix can be obtained as shown in

(3) $$\begin{array}{c} \left[\begin{array}{c} x_{0}\\ y_{0}\\ 1 \end{array}\right]=\left[\begin{array}{ccc} 1 & 0 & ‐t_{x}\\ 0 & 1 & ‐t_{1}\\ 0 & 0 & 1 \end{array}\right]\left[\begin{array}{c} x_{1}\\ y_{1}\\ 1 \end{array}\right]. \end{array}$$

It is shown in

(4) $$\begin{array}{c} \left\{\begin{array}{c} x_{0}=x_{1}-t_{x},\\ y_{0}=y_{1}-t_{y}. \end{array}\right. \end{array}$$

In this way, every point on the translated image can be found in the original image. For example, for the pixel (0, 0) in the new graph, substitute into the above equations, and the corresponding pixel (−*t*_*x*_, −*t*_*y*_) in the original graph can be obtained. If *t*_*x*_ or *t*_*y*_ is greater than 0, then (−*t*_*x*_, −*t*_*y*_) is not in the original image. For points that are not in the original image, you can simply set the pixel value to 0 or 255 (black or white for grayscale images). Similarly, if something is not in the original image, it means that something in the original image has been removed from the display area. If you do not want to lose part of the removed image, you can enlarge the width by |*t*_*x*_| and height of the newly generated image by |*t*_*y*_|. Changing the image mirror is divided into two types: one is horizontal glass and the other is vertical glass. The operation of the horizontal mirror of the image is to replace the left and right half of the image with the vertical line of the image. Vertical mirror work is the shape of the upper half and half of the image, with the horizontal axis of the image being the center of the mirror. Set the height of the image as height and width as width. After horizontal mirroring, the coordinates of (*x*_0_, *y*_0_) in the original image will change to (Width‐x_0_, y_0_}, and the matrix expression is shown in

(5) $$\begin{array}{c} \left[\begin{array}{c} x_{1}\\ y_{1}\\ 1 \end{array}\right]=\left[\begin{array}{ccc} -1 & 0 & \text{Width}\\ 0 & 1 & 0\\ 0 & 0 & 1 \end{array}\right]\left[\begin{array}{c} x_{0}\\ y_{0}\\ 1 \end{array}\right]. \end{array}$$

The expression of inverse operation matrix is shown in

(6) $$\begin{array}{c} \left[\begin{array}{c} x_{0}\\ y_{0}\\ 1 \end{array}\right]=\left[\begin{array}{ccc} -1 & 0 & \text{Width}\\ 0 & 1 & 0\\ 0 & 0 & 1 \end{array}\right]\left[\begin{array}{c} x_{1}\\ y_{1}\\ 1 \end{array}\right]. \end{array}$$

It is shown in

(7) $$\begin{array}{c} \left\{\begin{array}{c} x_{0}=\text{Width}-x_{1},\\ y_{0}=y_{1}. \end{array}\right. \end{array}$$

Similarly, the coordinate of (*x*_0_, *y*_0_) will change to (*x*_0_, Height‐*y*_0_) after vertical mirror image, and its matrix expression is shown in

(8) $$\begin{array}{c} \left[\begin{array}{c} x_{1}\\ y_{1}\\ 1 \end{array}\right]=\left[\begin{array}{ccc} 1 & 0 & 0\\ 0 & ‐1 & \text{Height}\\ 0 & 0 & 1 \end{array}\right]\left[\begin{array}{c} x_{0}\\ y_{0}\\ 1 \end{array}\right]. \end{array}$$

The expression of inverse operation matrix is shown in

(9) $$\begin{array}{c} \left[\begin{array}{c} x_{0}\\ y_{0}\\ 1 \end{array}\right]=\left[\begin{array}{ccc} 1 & 0 & 0\\ 0 & ‐1 & \text{Height}\\ 0 & 0 & 1 \end{array}\right]\left[\begin{array}{c} x_{1}\\ y_{1}\\ 1 \end{array}\right]. \end{array}$$

It is shown in

(10) $$\begin{array}{c} \left\{\begin{array}{c} x_{0}=x_{1},\\ y_{0}=\text{Height}-y_{1}. \end{array}\right. \end{array}$$

According to the above transformation formula, image horizontal and vertical mirror operation can be very simple. The following is the procedure flow chart of mirror operation, as shown in Figure 2:

The requirements of medical image processing system are analyzed, and the software development tools and development environment are introduced. Then, the whole frame of image processing is designed according to the functional requirements, and the function of each module in the frame is simply introduced. Then, according to the framework structure, the design of software is carried out. First, the user interface is designed according to the system framework. Then, according to the functions involved in the interface, the basic functional principles and program design ideas are described [14]. It focuses on the application and realization of image segmentation and pattern recognition in this software, which can be used as an auxiliary tool for doctor diagnosis.

The article "Application of CT Scan in Diagnosis of Iliac-Femoral Vein Thrombosis after Hip Replacement" was retracted in 2023. Reasons: signs of a paper mill; suspected computer-generated content; unreliable results or conclusions; lack of ethics approval or compliance.

## 4. Experiments and Analysis

Among the 90 patients under investigation, all of them completed the treatment without quitting during the course of treatment (the hospital stay of patients undergoing bone joint replacement is generally about 2 weeks, which is short and patients have good compliance) [15, 16]. There were 27 males and 63 females, with an average age of 20-883 years, with an average age of 52.45 ± 12.39. There are 32 patients with fractures in the neck, 51 patients with gynecological necrosis and osteoarthritis, and 7 patients with osteoarthritis of the bones and spine. There was no significant difference in the sex, age, and disease history of the patients (*P* > 0.05), as shown in Table 1:

At the end of the experiment, the number of patients with deep atherosclerosis in both groups was low. Diagnosis of atherosclerosis was confirmed by color Doppler ultrasound and was the rate of venous thrombosis in both groups. The control group had 6 patients, the incidence was 13.33070, and the intervention group had 0 patients, with a difference between the two groups (*P* = 0.034). The probability of intervention in the signature group (+) was 28.89%, and the difference was significant compared to the control group (*X*^2^ = 4.630, *P* = 0.031). The Neuhof mark (+) incidence in the intervention group was 22.220%, and the statistical difference was significant compared to the control group (*X*^2^ = 5.954, *P* = 0.015). The incidence of both the human mark (+) and the Neuhof mark (+) in the affected group was lower than that in the control group, with a significant difference (*P* < 0.05) as shown in Table 2.

The article "Application of CT Scan in Diagnosis of Iliac-Femoral Vein Thrombosis after Hip Replacement" was retracted in 2023. Reasons: signs of a paper mill; suspected computer-generated content; unreliable results or conclusions; lack of ethics approval or compliance.

The body surface temperature of 5 cm above the ankle of the two groups was measured and compared. It was found that there was no difference in the body surface temperature of the two groups before surgery, and the body surface temperature showed an upward trend after surgery and generally decreased gradually on the 7th day after surgery [17, 18]. On days 2, 3, 4, and 7 after surgery, the feet in the affected group had a body height of more than 5 cm lower than that of the body temperature control group (*P* < 0.05). On day 1, one day after surgery, 5 days after surgery, on day 6, day 8, and one day after surgery, the body temperature was 5 cm higher than the ankles of both groups (*P* > 0.05), as shown in Table 3.

The temperature changes of the two groups of patients were depicted by drawing, and it was intuitively found that the temperature of 5 cm above the ankle in both groups increased after surgery. The peak value was reached on the fourth day and then decreased, and the decline rate was consistent from the eighth day. The changes of body temperature at 5 cm above the ankle in the two groups showed that in the early postoperative period, the body temperature at 5 cm above the ankle in the intervention group was lower than that in the control group (*P* < 0.05), as shown in Figure 3.

The peak velocity and average velocity of femoral vein were detected before surgery and the 1st and 7th day after surgery for statistical analysis. The results showed that there was no significant change between the two groups before surgery, and there was no statistical difference (*P* > 0.05). One day after the first surgery, the control group was lower than the surgery, the response group was higher than the surgery, and the highest of the two groups was significantly higher (*P* > 0.05). But no difference was found in mean speed (*P* > 0.05) [19]. On the 7th day after the surgery, the peak and moderate flow rates of the two groups were higher than before the surgery, and the increase was more pronounced in the affected group. The differences between the two groups were significant (*P* < 0.05), as shown in Table 4.

Virchow proposed that the conditions of venous thrombosis need three factors: slow blood flow, damage to the vascular wall, and high blood coagulation state. Venous thrombosis requires a combination of at least two factors, neither of which alone can lead to thrombosis, and either of which can lead to thrombosis, especially slow blood flow and hypercoagulability. Virchow's theory has been clinically verified for more than half a century and tested by a variety of advanced technologies [20]. Many factors can lead to venous thrombosis after trauma, including pathogenic genes, hypercoagulability, cytokine interactions in inflammatory response, and immobilization [21]. At present, the research on the causes of venous thrombosis after trauma is not perfect, and active postoperative prevention is not given, and the problem of venous thrombosis after joint replacement is not sufficiently understood. Major orthopedic surgery, femoral shaft fracture, femoral neck fracture, and other operations, especially bone joint replacement, are prone to thrombosis in lower limb veins due to the long operation time and complicated operation process. During surgery, the body tissue and blood vessels are pulled for a long time, causing tissue damage and then activating the endogenous and exogenous coagulation system [22, 23]. After the coagulation system is started, the coagulation factors in the blood increase, while the operation causes damage to the intima of the blood vessel wall. Platelets attach to the damaged blood vessel wall, release bioactive substances, and promote the formation of thrombosis. During surgery, blood loss can lead to blood concentration, further exacerbating hypercoagulability. Elderly patients often combine with a variety of diseases, such as hyperlipidemia and hypertension. These illnesses can make the body enter the state of hypercoagulability. After surgery, the patient was weak and needed to stay in bed for a long time to slow down the venous return of the lower limbs. Therefore, more attention should be paid to the prevention of DVT in the elderly who undergo bone marrow transplantation. Once the DVT is established, the blood vessels can lead to loss of function, which not only reduces the quality of life of the patient but also worsens the patient, so prevention of DVT should be mentioned. Caring for patients with evidence of drug abuse refers to the process of planning the work of nursing staff in a nursing home, carefully considering and combining research findings with clinical and patient needs according to their needs. Perform the procedures. Evidence-based nursing practice has become a global consensus in nursing, and any professional decision in practice should be based on scientific evidence, not simply on experience. Bundles of care refer to a collection of therapeutic and nursing interventions that are based on evidence. It is aimed at the impact of many factors, difficult to solve the nursing problem. This nursing intervention is supported by evidence-based theory and was first proposed by the Institute for Healthcare Improvement (IHI). Its purpose is to help medical staff to provide better service, as far as possible to provide patients with more perfect and optimized medical and nursing services. This approach significantly reduces the incidence of DVT by combining evidence-based and effective measures for preventing DVT and maximizing the impact of these measures. Cluster nursing requires nursing staff to constantly sum up experience and lessons and grasp evidence-based evidence when implementing intervention measures. According to the original nursing evidence, give the best nursing plan, and in the nursing process, constantly improve the nursing basis and nursing plan. For patients with deep vein thrombosis, the main local symptoms are limb pain, heavy feeling of limbs, limb swelling, and tenderness (+). Sometimes, it can be accompanied by systemic symptoms, such as increased body temperature and accelerated heart rate; common signs are lower limb edema, skin pigmentation, ulcer, and other signs in severe cases. The larger and the lower limb thrombus, the more blocked blood flow, the slower the reflux, and the larger the swelling range. The faster the clot forms, the more pain the patient feels [24]. Distal venous thrombosis is slow, insidious, and usually undetected, with only mild pain in some patients. Or only the knee below the slight swelling of the limb, the disease further development, can appear Homan sign and Neuhof sign positive. Proximal venous thrombosis is rapid, the onset of acute, can quickly appear lower limb pain, accompanied by high fever and other systemic symptoms, and due to blood reflux disorder, can lead to obvious swelling of the lower limb, the affected side of the skin, subcutaneous weakness and subcutaneous venous expansion. Some blood vessels in the process of thrombosis, because thrombosis stimulates the blood vessel wall, can cause vascular spasm, aggravating the obstruction of blood return of patients with limb ischemia, severe pain, pale limbs, and other symptoms [25]. In clinical work, we found that most patients with venous thrombosis did not have typical symptoms, and the more common symptoms were limb swelling, increased skin temperature, and lower limb pain. Therefore, it is necessary to strengthen the comparison of lower limb swelling degree, temperature, and skin color to improve the early diagnosis rate. In this study, there were 6 cases of thrombosis in the red control group and no cases of thrombosis in the intervention group, and the difference between the two groups was statistically significant. Evidence-based cluster nursing intervention can effectively reduce lower extremity deep vein thrombosis after bone joint replacement. The main symptoms of venous thrombosis are local and systemic reactions. Iliac vein, femoral vein, and popliteal vein thrombosis often caused varying degrees of pain, swelling, and heaviness in the affected limbs. Sometimes, it can be accompanied by systemic symptoms, such as increased body temperature and accelerated heart rate; common signs are lower limb edema, skin pigmentation ulcer, and other signs in severe cases. Clinical common thrombosis is mostly a small range of thrombosis, thrombosis of small venous plexus generally has a small embolization range, the systemic reaction is relatively mild, generally only showing mild pain, and mild swelling of the side of the limb skin temperature slightly increased. This study showed that the postoperative surface temperature of the affected limbs showed an upward trend and generally decreased gradually on the 7th day after surgery. The body surface temperature of 5 cm limb above the ankle in the intervention group was significantly lower than that in the control group on the 2nd, 3rd, 4th, and 7th day after surgery (*P* < 0.05). The body temperature is 0 cm below the skeleton and 15 cm above the skeleton and is lower than that of the control group on the 1st, 2nd, 3rd, and 4th day after surgery. In this study, it was confirmed that evidence-based cluster nursing intervention could reduce the skin temperature of 5 cm above the ankle, 10 cm below the skeleton, and 15 cm above the skeleton of the affected limb 1–4 days after surgery. After surgery, due to postoperative bed rest, slow venous reflux, and other factors, mild swelling around the incision after surgery can be caused, which is mostly normal. If the patient develops edema of the limb and progresses from the distal to the proximal end of the limb, it is usually caused by venous stasis. When a thrombus forms in the venous tube, blood return is slowed and the distal venous return is blocked, causing the distal venous pressure to rise. Capillary filter pressure increased, coupled with anoxia and capillary permeability, and increased limb swelling. In venous thrombosis, the arteries spasm and lymphatic return is blocked, causing swelling of the limb in the affected area. Femoral vein thrombosis, resulting in blocked blood flow in the lower limb, blocked capillary flow, and tissue fluid cannot smoothly enter the vein, resulting in swelling of the knee or lower thigh limb. The results of this study showed that cluster nursing intervention could significantly reduce the limb circumference of 15 cm on the affected side of the body bones on the 3rd, 4th, and 5th day after surgery, but there was no significant difference in the limb circumference of 5 cm on the ankle [26, 27]. Evidence-based cluster nursing interventions can reduce limb swelling. After thrombosis of the muscle vein of the calf, certain physical stimulation can cause pain, especially in dorsiflexion of the ankle joint, the pain is more obvious, and this phenomenon is called Homan sign (+). If the patient has pain when pressing on the fat intestinal muscle, this is called Neuhof sign (+). The main mechanism is that the soleus muscle and fat intestine muscle are passively elongated at the dorsiflexion position of the ankle joint, which stimulates the diseased veins and causes limb pain. When distal deep vein thrombosis occurs in lower limbs, Homan sign and Neuhof sign can show positive signs, so Homan sign and Neuhof sign can be used as the examination to judge whether there is distal vein thrombosis. The results of this study show that compared to the control group, the positive characteristics of Homan and Neuhof in the group were slightly affected, with significant differences between the two groups. Evidence has shown that DVT can reduce the risk of a combination of surveillance services.

The article "Application of CT Scan in Diagnosis of Iliac-Femoral Vein Thrombosis after Hip Replacement" was retracted in 2023. Reasons: signs of a paper mill; suspected computer-generated content; unreliable results or conclusions; lack of ethics approval or compliance.

## 5. Conclusion

Iliac vein compression syndrome (IVCS) is also known as May-Thurner syndrome or Cockett syndrome. It refers to long-term compression of the right iliac artery in the anterior left iliac vein (LIV) of the lumbar spine with symptoms of deep iliac vein thrombosis (DVT) or venous hypertension such as swollen varicose veins in the left leg. It is associated with symptoms of atherosclerosis, such as deep atherosclerosis (DVT) or atherosclerosis in the left leg. Because of this relationship, many people have varying degrees of muscle contraction on the left side of the CT, but there are no signs of deep atherosclerosis or high blood pressure on the left side. Left lean muscle compression during CT scan is not the same as general lean muscle compression disease. Diagnosing the syndrome of atherosclerosis requires three components. First, the left ventricle is compressed by the right artery. Second, the angiography of the arteries shows that the air sac is thin and narrow and that a large artery can be seen in the abdominal cavity. Third, there is clinical evidence of deep atherosclerosis or intravenous hypertension, such as atherosclerosis or lower limb inflammation. Fourth, treatment occurs at the lower extremities of the arteries, such as at the lower extremities or at the lower extremities, or at the lower right atrium. Complications of pulmonary embolism are very rare. Foreign data has now been reported in right-hand muscle contractions. Fretz reported abnormal contractions of the right muscle due to a split in the pancreas, resulting in a narrowing of the inferior vena cava through most of the pelvic floor muscles and the right artery. Abboud and Burkespierre reported narrowing of the right artery from the right artery due to differences in the veins on the left. All of the above 3 conditions for right-hand muscle contraction have vascular changes. Molloy reports data on right-sided muscle contraction syndrome, in which the right muscle is compressed by the right internal artery, but the lower extremity and CT images are missing. The study reported that right-sided vascular compression syndrome was reported without modifying the blood vessels and that the patient's treatment of low blood pressure (e.g., lower limb arteries) was suggested. Lower venous arteries indicate severe pain in the arteries and many arteries in the abdomen. CT scan shows that the right atrium is constricted by the right artery. Some studies have shown that compression of the coronary artery disease and deep vein congestion of the lower left leg are more common in women. Malignant neoplasms are more common in men. This is because in the development of lumbar spine in women, the lumbar spine rises forward, increasing the risk of muscle spasms on the left side. This is because in the development of lumbar spine in women, the lumbar spine rises forward, increasing the risk of muscle spasms on the left side. During the three months, lumbar spine disease also increases, so the contraction of the left intestinal muscle becomes more pronounced in the third trimester and after childbirth, which increases the risk of DUT in the lower left. In this study, men had more muscle contraction on the right side than women, and women had more muscle contraction on the left than men. The number of female patients with left ventricular compression is >50% higher than in men. These are anatomical features that describe the different sexes in the DUT that occur on the right and left.

The article "Application of CT Scan in Diagnosis of Iliac-Femoral Vein Thrombosis after Hip Replacement" was retracted in 2023. Reasons: signs of a paper mill; suspected computer-generated content; unreliable results or conclusions; lack of ethics approval or compliance.

## Figures and Tables

**Figure 1:** CT application of microscope scanning in diagnosis of iliac-femoral vein thrombosis after hip replacement.

**Figure 2:** Flowchart of image mirroring program.

**Figure 3:** Comparison of temperature of 5 cm upper ankle limb between the two groups.

**Table 1:** General patient information.

Project		Control group (*n* = 45)	Intervention group (*n* = 45)	*t*/*X*^2^	*P*
Number of cases		45 (constituent ratio)	45 (constituent ratio)		
Sex	Male	13 (28.98%)	14 (32.33%)	0.053	0.818
	Female	32 (71.11%)	31 (68.89%)		
Education	Junior high and below	31 (68.89%)	29 (64.44%)	0.200	0.655
	Junior high and above	14 (31.11%)	16 (35.56%)		
Replacement parts	Left	18 (40.00%)	19 (42.22%)	0.118	0.943
	Right	21 (46.67%)	21 (46.67%)		
	Two sides	6 (13.33%)	5 (11.11%)		
Material type	Biological type	24 (53.33%)	27 (60.00%)	0.407	0.523
	Bone cement type	21 (46.67%)	18 (40.00%)		
Hypertension		17 (37.78%)	15 (33.33%)	0.194	0.660
Diabetes		11 (24.44%)	10 (22.22%)	0.062	0.803
Varicosity		12 (26.67%)	10 (22.22%)	0.241	0.624
Age		6233 ± 6.58	61.12 ± 7.08	O.840^∗^	0.403
BMI (kg/m^2^)		24.85 ± 3.08	24.35 ± 3.11	0.766^∗^	0.446
Operation time (min)		125 ± 32.05	128.11 ± 30.18	-0.474^∗^	0.637

**Table 2:** Comparison of venous thrombosis and Homan sign (+) and Neuhof sign (+) between the two groups.

Group	*n*	Homan sign (+)	Neuhof sign (+)	Deep vein thrombosis of the lower extremity (%)
Control group	45	23	21	6 (13.33%)
Intervention group	45	13	10	0 (0.00%)
*X* ^2^		4.630	5.945	4.460
*P*		0.031^a^	0.015^a^	0.034^b^

**Table 3:** Comparison of the temperature of 5 cm upper ankle limb between the two groups (*x* ± *s*, °C).

Group	*n*	Preoperative	Postoperative day 1	Postoperative day 2	Postoperative day 3	Postoperative day 4
Control group	45	33.49 ± 1.49	33.95 ± 0.82	35.85 ± 1.02	35.48 ± 0.55	35.39 ± 0.75
Intervention group	45	33.46 ± 1.56	33.65 ± 1.01	34.94 ± 0.57	34.70 ± 0.88	34.99 ± 0.96
*t*		0.093	1.547	5.224	5.042	2.203
*P*		0.926	0.125	0.000	0.000	0.030

**Table 4:** Comparison of peak and average velocity of femoral vein between two groups.

Group	*n*	Preoperative		Postoperative day 1		Postoperative day 7	
		Peak systolic velocity	Mean flow rate	Peak systolic velocity	Mean flow rate	Peak systolic velocity	Mean flow rate
Control group	45	17.01 ± 2.78	12.01 ± 3.03	16.32 ± 3.15	11.86 ± 3.71	20.01 ± 3.57	13.91 ± 3.26
Intervention group	45	16.78 ± 3.47	11.68 ± 3.01	17.89 ± 4.01	12.01 ± 4.15	25.10 ± 4.79	15.75 ± 3.02
*t*		0.347	0.518	-2.065	-0.181	-5.716	-2.778
*P*		0.729	0.606	0.042	0.857	0.000	0.007

## Data Availability

The data used to support the findings of this study are available from the corresponding author upon request.
